The article "MicroRNA-338-3p suppresses ovarian cancer cells growth and metastasis: implication of Wnt/catenin beta and MEK/ERK signaling pathways" was retracted in 2024. Reasons: duplicated images; unreliable results or conclusions; concerns about the data.

# MicroRNA-338-3p suppresses ovarian cancer cells growth and metastasis: implication of Wnt/catenin beta and MEK/ERK signaling pathways

**DOI:** 10.1186/s13046-019-1494-3

**Published:** 2019-12-16

**Authors:** Ruitao Zhang, Huirong Shi, Fang Ren, Wei Feng, Yuan Cao, Gailing Li, Zheying Liu, Pengcheng Ji, Minghui Zhang

**Affiliations:** Department of Gynecology, First Affiliated Hospital, Zhengzhou University, NO.1 East Jianshe Road, Erqi District, Zhengzhou, Henan 450052 People’s Republic of China

**Keywords:** miR-338-3p, Ovarian cancer, MACC1, Met, Growth, Metastasis

## Abstract

**Background:**

Downregulation of microRNA-338-3p (miR-338-3p) was detected in many malignant tumors, which indicated miR-338-3p might serve as a role of antioncogene in those cancers. The present study aimed to explore the roles of miR-338-3p in the growth and metastasis of ovarian cancer cells and elaborate the underlying possible molecular mechanism.

**Methods:**

Multiply biomedical databases query and KEGG pathway enrichment assay were used to infilter possible target genes and downstream pathways regulated by miR-338-3p. Overexpression miR-338-3p lentiviral vectors were transfected into ovarian cancer OVCAR-3 and OVCAR-8 cells, cell proliferation, migration and invasion were analyzed by MTT, colony formation, transwell, Matrigel assay and xenograft mouse model. One 3′-untranslated regions (UTRs) binding target gene of miR-338-3p, MACC1 (MET transcriptional regulator MACC1), and its regulated gene MET and downstream signaling pathway activities were examined by western blot.

**Results:**

Biomedical databases query indicated that miR-338-3p could target MACC1 gene and regulate Met, downstream Wnt/Catenin beta and MEK/ERK pathways. Rescue of miR-338-3p could inhibit the proliferation, migration and invasion of ovarian cancer cells, and suppress the growth and metastasis of xenograft tumor. Restoration of miR-338-3p could attenuate MACC1 and Met overexpression induced growth, epithelial to mesenchymal transition (EMT) and activities of Wnt/Catenin beta and MEK/ERK signaling in vitro and in vivo.

**Conclusions:**

The present data indicated that restoration of miR-338-3p could suppress the growth and metastasis of ovarian cancer cells, which might due to the inhibition of proliferation and EMT induced by MACC1, Met and its downstream Wnt/Catenin beta and MEK/ERK signaling pathways.

## Background

Sustaining proliferative signaling and activating invasion and metastasis are two important malignant hallmarks of human cancer [1], which also can be observed in ovarian cancer,especially in advanced ovarian cancer. Extensive disseminated growth and distant metastasis in the pelvic and abdominal cavity are the most important malignant biological characteristics of advanced ovarian cancer. Target therapy, cell cycle regulator and immunotherapy methods, like PARP and CDK4/6 inhibitors and PD-1 or PD-L1 antibodies, are effective complements of Platinum-based combination chemotherapy after cytoreductive surgery and new exciting therapeutic ways to prolong the survival time for chemoresistance and recurrence ovarian cancer patients [2–4]. However, ovarian cancer still is the most lethal gynecological malignancy [5]. Inhibition of malignant abilities, like endless proliferation and activating invasion and metastasis, seems to be the fundamental way to solve this troublesome problem in ovarian cancer. Therefore, explore the molecular mechanism of malignant growth and metastasis might provide new therapy strategies for ovarian cancer.

The article "MicroRNA-338-3p suppresses ovarian cancer cells growth and metastasis: implication of Wnt/catenin beta and MEK/ERK signaling pathways" was retracted in 2024. Reasons: duplicated images; unreliable results or conclusions; concerns about the data.

MicroRNAs (miRNAs), earliest discovered non-coding RNAs, are well demonstrated to be implicated in the cell proliferation, invasion and metastasis of almost all types of human cancers [6]. Emerging evidences showed upregulation of miR-338-3p could target different downstream genes and signaling pathways to inhibit malignant cells proliferation, migration and invasion in rectal cancer, gastric cancer, lung cancer, neuroblastoma and liver cancer, which indicated miR-338-3p might be associated with the initiation and progression of these human cancers [7–11]. Only few researches involved in the relation between miR-338-3p and ovarian cancer. One study indicated miR-338-3p could inhibit the proliferation and metabolism of ovarian cancer, and the other showed miR-338-3p could suppress growth of ovarian epithelial carcinoma cells by targeting Runx2 [12, 13]. We previously reported miR-338-3p was decreased and negatively related with MACC1 (MET transcriptional regulator MACC1) in epithelial ovarian cancer tissues [14]. Thence, the roles of miR-338-3p involved in ovarian cancer still need more research.

In present study, we overexpressed miR-338-3p, MACC1, one 3′-untranslated regions (UTRs) binding target gene of miR-338-3p, and its regulated gene MET in ovarian cancer cells respectively to explore the effects on proliferation, epithelial to mesenchymal transition (EMT) and downstream pathways in vitro and in vivo, and to elaborate the roles of miR-338-3p in the growth and metastasis of ovarian cancer.

## Methods

### Biomedical database query

Multiply biomedical databases, including dbDEMC [15], cBioPortal [16], OncomiR [17], miRTargetLink [18], TargetScan Human [19], microT-CDS [20], miRpathDB [21] and miRTarBase [22] were queried to examine the expressions of miR-338-3p in ovarian cancer tissues and to filter its possible target genes.

The article "MicroRNA-338-3p suppresses ovarian cancer cells growth and metastasis: implication of Wnt/catenin beta and MEK/ERK signaling pathways" was retracted in 2024. Reasons: duplicated images; unreliable results or conclusions; concerns about the data.

### KEGG pathways enrichment analysis

ENCORI database (Previous version named starBase database, http://starbase.sysu.edu.cn/) was used to perform Kyoto Encyclopedia of Genes and Genomes (KEGG) pathways enrichment analysis for miR-338-3p, MACC1 and Met to filter downstream regulation pathways.

### Cell culture and reagents

The ovarian cancer cell lines SKOV3, OVCAR3 and A2780 were obtained from China Center for Type Culture Collection (CCTCC) and OVCAR8 cells were obtained from American Type Culture Collection (ATCC), which were cultured in DMEM or RPMI 1640 medium. Immortalized human ovarian epithelial cells SV40 were obtained from Applied Biological Materials Inc. (Richmond, Canada) and cultured in Prigrow I medium (Abm, Richmond, Canada). Mentioned cell culture mediums were supplemented with 10% fetal bovine serum (FBS) and 1% Penicillin/Streptomycin (Hyclone; Logan, UT). HEK293FT cells were purchased from Thermo Fisher Scientific Inc. (Waltham, Massachusetts, USA) and cultured in DMEM medium with 10% FBS, 0.1 mM non-essential amino acids, 6 mM L-glutamine, 1 mM Sodium Pyruvate and 1% Pen-Strep. All cells were maintained in 5% Carbon dioxide, 37.0 °C and 95% humidity incubator. Cells were cleared of mycoplasma contamination.

Wnt/Catenin beta signaling inhibitor IWP-2 and MEK/ERK signaling inhibitor UO126 were purchased from Beyotime Biotechnology (Shanghai, China).

### Lentiviral vectors and cell transfection

Lentiviral miRNA control vectors, which were used to construct miR-338-3p overexpression lentivectors and were sequenced by RiboBio (Guangzhou, China), MACC1 and Met overexpression and control lentivectors were obtained from Abm Inc. (Richmond, Canada). All lentivectors were packaged in HEK293FT cells by lentivirus packaging mix (Abm, Richmond, Canada) following the protocol of manufacturer. Lentivectors were purified and transfected into OVCAR3 and OVCAR8 cells with polybrene, stable pools of transfected cells were selected with 5 μg/ml puromycin.

### Real time PCR

Cell total RNA were isolated by Trizol reagent (Invitrogen, Carlsbad, Calif., USA), 2 μg total RNA were used to reverse-synthesize cDNA template following the TaqMan MicroRNA Reverse Transcription kit instructions (Applied Biosystems Co., Ltd. USA) for SYBR Green PCR (Takara, Dalian, China) assay. The PCR primers and reaction conditions were produced as described previously, and expression of miR-338-3p was normalized to U6 [14]. Each PCR experiment was performed for three times independently, and the relative expression value was expressed by 2^-ΔΔCt^ method.

### Western blot

The antibodies used in Western blot assay were glyceraldehyde 3-phosphate dehydrogenase (GAPDH, AF0006), Met (AF0120), proliferating cell nuclear antigen (PCNA, AF0261), MMP2 (AF0234), E-cadherin (AF0138), Cytokeratin7 (AF0129), N-cadherin (AF0243), Vimentin (AF0318), Catenin beta (AF0069), t-MEK1/2 (AF1057),p-MEK1 (AF1786), t-ERK1/2 (AF1051), p-ERK1/2 (AM071) (Beyotime Biotechnology, Shanghai, China), and MACC1 (86,290 s), MMP9 (13,667 s), Wnt3a (2391s), p-LRP6 (2568s), LRP6 (3395s) (Cell Signaling, Danvers, USA). Total protein was collected by RIPA buffer (Beyotime Biotechnology, Shanghai, China) containing proteinase inhibitor, equal amount of protein (50 μg per lane) was used to perform 8–10% SDS-PAGE separation and immunoblot as described previously [23].

The article "MicroRNA-338-3p suppresses ovarian cancer cells growth and metastasis: implication of Wnt/catenin beta and MEK/ERK signaling pathways" was retracted in 2024. Reasons: duplicated images; unreliable results or conclusions; concerns about the data.

### Dual-luciferase reporter assay

Wild type and mutant type MACC1 3’UTR binding sites of hsa-miR-338-3p were cloned into pMIR-GLO™ Dual-Luciferase miRNA Target Expression Vector (Promega, Madison, WI, USA) by RiboBio (Guangzhou, China). OVCAR3 and OVCAR8 cells were planted into 96-well plate in triplicate for 24 h, and co-transfected with wild type or mutant type MACC1 3’UTR vectors together with miR-338-3p overexpression or control lentivectors. After incubation for another 48 h, luciferase activities were measured using dual-luciferase reporter assay system (Promega, Madison, WI, USA) following the manufacturer’s protocol. Renilla luciferase activities were used as normalization.

### MTT assay

Planted 1 × 10^4^ cells per well into 96-well plates, five duplicate wells were set up for each group. Cultured cells continuously for 3 days, added 20 μl MTT reagent (5 mg/mL, Sigma, St. Louis, USA) into each well, incubated for another 4 h then aspirated former medium and added 150 μl DMSO. The absorbances of sample were measured by Microplate spectrophotometer (Thermo, Spectronic, Madison, WI, USA) at 492 nm.

### Cell colony formation assay

Cells (300 per well) were plated into 6-well plate in triplicate for 10 days culturation, stained cells with 0.1% Crystal Violet after fixation in methanol for 20 min, and cell colonies with more than 50 cells were counted using Image J software.

### Cell migration assay

Cells were pretreated with serum free medium for 24 h, 3 × 10^5^ cells in 300 μl serum free medium were added into the upper transwell chamber (BD Falcon, San Jose, CA). 700 μl medium with 10% FBS was added into each well where the chambers were inserted. After incubation for another 16 h, the chamber membranes were fixed with methanol for 20 min and stained with crystal violet for 15 min. Cells on the lower membranes in at least three different fields were counted under 10× magnification.

### Cell invasion assay

Except for the following steps, other processes were the same as the transwell migration assay. Chambers used for invasion assay were precoated with Matrigel (BD BioCoat), cells were incubated for another 36 h after planting,and the transwell inserts were stained by H&E method.

The article "MicroRNA-338-3p suppresses ovarian cancer cells growth and metastasis: implication of Wnt/catenin beta and MEK/ERK signaling pathways" was retracted in 2024. Reasons: duplicated images; unreliable results or conclusions; concerns about the data.

### Mouse xenograft model

Animal experiment protocols were approved by the ethics committee of the first affiliated hospital of Zhengzhou University. Eight two-month-old female NOG(NOD.Cg-Prkdc^scid^Il2rg^tm1Sug^/JicCrl)mice (Charles River, Beijing, China) were randomly divided into two groups with four mice in each group. Control and stable miR-338-3p overexpression lentivectors transfected OVCAR-8 cells (1 × 10^6^ cells in 10 μl PBS per mouse) labeled with luciferase lentivectors were injected into the left ovary after Isoflurane inhalation anesthesia. Tumor initiation and progression were monitored once a week using an IVIS Spectrum system (Xenogen, Caliper Life Sciences). All mice were sacrificed at the fourth week after cell inoculation.

### Immunohistochemistry

Xenograft tumor tissues were fixed in formalin, embedded in paraffin and sectioned at 3 μm for immunohistochemistry assay. Expressions of MACC1, Met, PCNA, E-cadherin and Catenin beta were detected by broad spectrum immunohistochemistry SP kit and metal enhanced DAB substrate kit (Solarbio, Beijing, China) following manufacture’s protocol. Protein relative positive ratios were measured by Image J software in at least three independent fields.

### Statistical analysis

Significant differences were determined with one-way analysis of variance (one-way ANOVA) and Student’s t-test by SPSS 21.0 and GraphPad Prism 7.0 software packages, data were presented as mean ± SD. *P*-values less than 0.05 were regarded as statistically significant, while the values ^**^ *P* < 0.01 and ^***^ *P* < 0.001 were considered to indicate increased statistical significance.

## Results

### miR-338-3p was downregulated in ovarian cancer tissues and could target MACC1

The expression profiles of miR-338-3p in ovarian cancer queried in multiply biomedical databases well confirmed to our previous report [14]. Compared to 7 cases normal fallopian samples, miR-338-3p and other 174 miRNAs were decreased in 114 high-grade and advanced stage epithelial ovarian, primary peritoneal or fallopian tube serous carcinoma tissue samples detected by whole-genome characterization assay (Fig. 1a). In three independent TCGA cohort data with total 1680 ovarian serous adenocarcinoma tissue samples, most samples could not detect miR-338-3p alteration, 4 cases detected deep deletions, and only 69 cases detected amplifications, which also showed an expression profile negative related to MACC1 (Fig. 1b,c). Down-regulations of miR-338-3p in ovarian cancer tissues were also detected in OncomiR database (Fig. 1d). These data showed expression profile of miR-338-3p was downregulated in ovarian cancer tissues.

The article "MicroRNA-338-3p suppresses ovarian cancer cells growth and metastasis: implication of Wnt/catenin beta and MEK/ERK signaling pathways" was retracted in 2024. Reasons: duplicated images; unreliable results or conclusions; concerns about the data.

**Fig. 1:** Expressions of miR-338-3p in ovarian cancer tissues and possible target genes queried by multiply biomedicial databases. **a** Differential expression profile of miR-338-3p in cancer vs normal tissues shown in dbDEMC database; **b** Expressions of miR-338-3p and MACC1 in three TCGA cohorts indicated by cBioPortal database; **c** Alteration frequency of miR-338-3p in three TCGA cohorts unfolded by cBioPortal database; **d** Serveral cancer related miRNAs expression profiles in human cancers explored in OncomiR database; **e** Target genes of miR-338-3p with strong supports showed by miRTargetLink database; **f** Venn diagram for target genes of miR-338-3p infiltered by TargetScan Human, microT-CDS, miRpathDB and miRTarBase databases interactive verification; **g** Input informations (Additional file 2) and output results of Venn diagram producer

MACC1 was 1 of 15 target genes of miR-338-3p with strong support showed by miRTargetLink database (Fig. 1e). Based on multiply database interactive verification, miR-338-3p could bind to the 3′- UTRs of MACC1 and MACC1 was one of downstream target genes of miR-338-3p (Fig. 1f,g, Additional file 2) which was also demonstrated by several independent reports in different cancer cells using dual-luciferase reporter assay or biotin-avidin pull-down assay [24–29]. Therefore, MACC1 should be one of downstream target genes of miR-338-3p.

### miR-338-3p could regulate met, Wnt/catenin beta and MEK/ERK pathways

Indicated by mir-Tar-pathway analysis in ENCORI database, miR-338-3p could regulate 328 genes of KEGG pathways in cancer (log10 FDR: − 9.52602, log10 *p* value: − 11.79554), including MET, WNT3A, CTNNB1 (Catenin beta), MAP2K1 (MEK1), MAP2K2 (MEK2), MAPK1 (ERK2), MAPK3 (ERK1), MMP2, MMP9 and CDH1 (E-cadherin). When referred to rna-Tar-pathway analysis, MET could regulate 75 genes of KEGG adherens junction pathways (log10 FDR: − 1.65161, log10 *p* value: − 3.23139), including MAPK1 (ERK2), MAPK3 (ERK1), CTNNB1 (Catenin beta) and CDH1 (E-cadherin). More detail data were shown in Additional file 1. These data indicated miR-338-3p could regulate Met, Wnt/Catenin beta and MEK/ERK pathways.

### miR-338-3p was decreased in ovarian cancer cells

To confirm the expression profiles in ovarian cancer tissues, expressions of miR-338-3p were examined in different ovarian cancer cells by real time PCR in present study. Compared to normal ovary epithelial cells, downregulated miR-338-3p was detected in ovarian cancer SKOV3, OVCAR3, A2780 and OVCAR8 cells (Fig. 2a) which indicated the expression profile of miR-338-3p was also decreased in ovarian cancer cells.

The article "MicroRNA-338-3p suppresses ovarian cancer cells growth and metastasis: implication of Wnt/catenin beta and MEK/ERK signaling pathways" was retracted in 2024. Reasons: duplicated images; unreliable results or conclusions; concerns about the data.

**Fig. 2:** Expressions of miR-338-3p in different ovarian cancer cells and confirmation of lentivectors transfection. **a** Expressions of miR-338-3p in normal ovary epithelial cells and different ovarian cancer cells examined by RT-PCR; **b** Expressions of miR-338-3p in blank, control and miR-338-3p overexpression lentivectors transfected OVCAR3 and OVCAR8 cell examined by RT-PCR; **c** Expressions of MACC1 and Met in blank, control and MACC1 overexpression lentivectors transfected OVCAR3 and OVCAR8 cell examined by western blot; **d** Expressions of MACC1 and Met in blank, control and Met overexpression lentivectors transfected OVCAR3 and OVCAR8 cell examined by western blot; **e** The wild type (Wt) MACC1 3′-UTR sequences and binding sites to miR-338-3p, and the mutant type (Mut) MACC1 3′-UTR sequences; **f** Relative luciferase activities measured by dual-luciferase reporter assay in OVCAR3 and OVCAR8 cells; **g** Expressions of MACC1 and Met in blank, control and miR-338-3p overexpression lentivectors transfected OVCAR3 and OVCAR8 cell examined by western blot

### Confirmation of lentiviral vectors transfection effects in ovarian cancer cells

Before malignant behavior assay, lentivectors transfection consequences were confirmed firstly. After 72 h puromycin treatment, total mRNA and protein of stable transfection cells were isolated for analysis. Compared to blank cells and control lentivectors transfected cells,levels of miR-338-3p were significantly upregulated after overexpression vectors transfection (Fig. 2b). Furthermore, MACC1 and Met overexpression lentivectors transfection effectively elevated MACC1 and Met levels in ovarian cancer cells respectively (Fig. 2c, d).

### miR-338-3p could directly target MACC1 in ovarian cancer cells

To confirm the direct interaction between miR-338-3p and MACC1, we performed dual-luciferase reporter assay following co-transfection wild type and mutant type MACC1 3′-UTR vectors with miR-338-3p overexpression or control lentivectors (Fig. 2e) in ovarian cancer cells. In OVCAR3 and OVCAR8 cells, lower luciferase activities were observed in wild type MACC1 3′-UTR and miR-338-3p overexpression vectors co-transfected cells compared with mutant type, which indicated mutation of the target site in the MACC1 3′-UTR abolished the inhibition of luciferase activity by miR-338-3p (Fig. 2f). Furthermore, expressions of MACC1 and Met were obviously downregulated after miR-338-3p overexpression in ovarian cancer cells (Fig. 2g). Therefore, our data confirmed that MACC1 was one directly target gene of miR-338-3p in ovarian cancer cells.

The article "MicroRNA-338-3p suppresses ovarian cancer cells growth and metastasis: implication of Wnt/catenin beta and MEK/ERK signaling pathways" was retracted in 2024. Reasons: duplicated images; unreliable results or conclusions; concerns about the data.

### Restoration of miR-338-3p inhibited the proliferation of ovarian cancer cells

Cell proliferation OD values and cell colony numbers decreased after miR-338-3p restoration in ovarian cancer cells. MACC1 or Met overexpression could increase cell proliferation OD values and cell colony numbers, but those proliferation promotive effects could be attenuated by miR-338-3p overexpression, at least partially (Fig. 3), which showed miR-338-3p could inhibit the proliferation of ovarian cancer cells induced by MACC1 and Met overexpression.

**Fig. 3:** Restoration of miR-338-3p inhibited the proliferation of ovarian cancer cells. Cell proliferation detected by MTT assay **a** and colony formation assay **b** in control, miR-338-3p overexpression, MACC1 overexpression, Met overexpression, miR-338-3p overexpression + MACC1 overexpression and miR-338-3p overexpression + Met overexpression lentivectors transfected OVCAR3 and OVCAR8 cells respectively

### Restoration of miR-338-3p suppressed the migration and invasion of ovarian cancer cells

Compared to control cells, decreased migration and invasion cell numbers were observed in transwell assay after rescue of miR-338-3p. MACC1 or Met overexpression could increase migration and invasion cell numbers, which also could be restrained following miR-338-3p overexpression (Fig. 4). Weakened aggressive cell phenotypes were also observed in miR-338-3p restoration cells (Fig. 5) in vitro. These data indicated miR-338-3p could suppress the migration and invasion abilities of ovarian cancer cells.

**Fig. 4:** Restoration of miR-338-3p suppressed the migration and invasion of ovarian cancer cells. Cell migration **a** and invasion **b** examined by transwell assay in control, miR-338-3p overexpression, MACC1 overexpression, Met overexpression, miR-338-3p overexpression + MACC1 overexpression and miR-338-3p overexpression + Met overexpression lentivectors transfected OVCAR3 and OVCAR8 cells respectively

**Fig. 5:** Restoration of miR-338-3p attenuated cell aggressive phenotypes in ovarian cancer cells. About 1 × 10^3^ cells per well were seeded into 6-well plate and cultured with 10% FBS for 48 h, cell phenotypes were captured under 40× magnification using a Nikon digital inverted microscope

### Restoration of miR-338-3p repressed xenograft tumor growth and metastasis

Before ovarian cancer cells inoculated mice sacrifice, the intensities of luminescence were measured for the last time. Compared to control cells induced tumors, the intensities of luminescence in miR-338-3p overexpression cells induced xenograft tumor were obviously decreased (Fig. 6a), as well as the tumor weights (Fig. 6b), which showed miR-338-3p enabled an inhibitory effect on the ovarian cancer cells induced tumor growth. Attenuated aggressiveness and metastasis of ovarian cancer cells were also observed in the ovary, liver and spleen tissue H&E staining sections of miR-338-3p restored mice tumors (Fig. 6c). These data suggested miR-338-3p could repress the growth and metastasis of ovarian cancer cell xenograft tumors.

The article "MicroRNA-338-3p suppresses ovarian cancer cells growth and metastasis: implication of Wnt/catenin beta and MEK/ERK signaling pathways" was retracted in 2024. Reasons: duplicated images; unreliable results or conclusions; concerns about the data.

**Fig. 6:** Restoration of miR-338-3p repressed xenograft tumor growth and metastasis. **a** The intensities of luminescence in control and miR-338-3p overexpression OVCAR8 cells induced mice xenograft tumors; **b** The weights of sacrificed mice left ovary xenograft tumors; **c** Xenograft tumor and metastasis tumor observed in the ovary, liver and spleen tissue H&E staining sections from mice xenograft model

### Restoration of miR-338-3p restrained MACC1 and met induced proliferation and EMT in vitro

Furthermore, we explored the possible mechanism of miR-338-3p induced inhibition of ovarian cancer cells growth and metastasis. Due to the recovery of miR-338-3p expression, MACC1 and Met expressions were downregulated in ovarian cancer cells. Upregulations of MACC1 or Met induced by MACC1 or Met overexpression lentivectors transfection could be attenuated when transfected miR-338-3p overexpression lentivectors simultaneously into ovarian cancer cells (Fig. 7a-b). Cell proliferation and EMT related proteins were also measured to explore the roles of miR-338-3p in cell proliferation and EMT. After restoration of miR-338-3p, expressions of PCNA, MMP2 and MMP9 (also two target genes of miR-338-3p indicated by miRTargetLink database, Fig. 1e) were downregulated, as well as the expressions of N-cadherin, Vimentin and Catenin beta, while expressions of E-cadherin and Cytokeratin7 were upregulated. Furthermore, MACC1 or Met overexpression could induce downregulations of E-cadherin and Cytokeratin7, and upregulations of PCNA, MMP2, MMP9, N-cadherin, Vimentin and Catenin beta, but could be attenuated by the restoration of miR-338-3p (Fig. 7a-d). Therefore, miR-338-3p could restrain the proliferation and EMT of ovarian cancer cells induced by MACC1 and Met overexpression.

**Fig. 7:** Restoration of miR-338-3p restrained growth, EMT, Wnt and MEK signaling in vitro. **a-d** Expressions of MACC1, Met, proliferation related marker PCNA, and EMT related markers E-cadherin and Cytokeratin7, N-cadherin, Vimentin, Catenin beta, MMP2 and MMP9 in control, miR-338-3p overexpression, MACC1 overexpression, Met overexpression, miR-338-3p overexpression + MACC1 overexpression and miR-338-3p overexpression + Met overexpression lentivectors transfected OVCAR3 and OVCAR8 cells respectively. **e-h** Activities of Wnt/Cadherin beta and MEK/ERK pathways examined by western blot in different groups, Wnt signaling inhibitor (30 μM IWP-2) and MEK signaling inhibitor (1 μM UO126) were used to treat control, MACC1 overexpression and Met overexpression cells for 24 h as a positive control

The article "MicroRNA-338-3p suppresses ovarian cancer cells growth and metastasis: implication of Wnt/catenin beta and MEK/ERK signaling pathways" was retracted in 2024. Reasons: duplicated images; unreliable results or conclusions; concerns about the data.

### Restoration of miR-338-3p inhibited the activities of Wnt and MEK signaling induced by MACC1 or met overexpression in vitro

Based on KEGG pathway assay, we detected the activities of canonical Wnt/Catenin beta and MEK/ERK pathways. As consequences of MACC1 or Met overexpression, levels of Wnt3a and p-LRP6, p-MERK1/2 and p-ERK1/2 were elevated, which could be attenuated by Wnt signaling inhibitor IWP-2 and MEK signaling inhibitor UO126 treatment respectively. Similar inhibitory effects were observed in control, MACC1 and Met overexpressed ovarian cancer cells following miR-338-3p restoration, which indicated miR-338-3p could attenuate MACC1 or Met induced Wnt and MEK signaling activities, at least in partially (Fig. 7e-h).

### Restoration of miR-338-3p suppressed proliferation, EMT, Wnt and MEK signaling in vivo

Total mRNA and protein from xenograft tumor tissues were also extracted after animal sacrifice. Upregulations of miR-338-3p, E-cadherin and Cytokeratin7, downregulations of MACC1, Met, PCNA, MMP2, MMP9, N-cadherin, Vimentin, Catenin beta, p-MEK1/2, p-ERK1/2, Wnt3a and p-LRP6 were detected respectively in miR-338-3p restoration cells injected mice tumor tissues compared to control cells injected mice tumor tissues (Fig. 8a-e). Expressions of MACC1, Met, PCNA, E-cadherin and Catenin beta in xenograft tumors were also confirmed by tissue section immunohistochemistry assay (Fig. 8f). These data suggested miR-338-3p could suppress the proliferation, EMT, Wnt and MEK signaling in xenograft tumor tissues.

**Fig. 8:** Restoration of miR-338-3p suppressed growth, EMT, Wnt and MEK signaling in vivo. **a**-**e** Total mRNA and protein samples isolated from every xenograft mouse tumor were used to perform RT-PCR and western blot assay; **f** Expressions of MACC1, Met, PCNA, E-cadherin and Catenin beta in xenograft tumor tissue sections were measured by immunohistochemistry method respectively

## Discussion

Based on the progresses of understanding the biology of human cancer, other well-known human cancer hallmarks are considered to collaborate to ensure tumor cells growth and metastatic dissemination [1]. Endless proliferation enables enough cell numbers to escape from the elimination of the body protection systems, and distant metastasis not only bases on enough cancer cell numbers but also provides new places for malignant cell growth. Both the two aggressive behaviors distinctively characterize cancer cells different with normal cells. When refers to ovarian cancer, malignant growth to distant metastasis to cytoreductive surgery to resurrected growth to uncontrollable metastasis seems to be a lethal cycle suffered most of ovarian cancer patients, especially for advanced stage strugglers. In past decades, many progresses have been observed in the biology research of ovarian cancer, including growth, apoptosis, autophagy, invasion, metastasis, metabolism, and angiogenesis [30, 31]. However, the molecular mechanisms underlying aggressive growth and metastasis of ovarian cancer cells still need further study.

The article "MicroRNA-338-3p suppresses ovarian cancer cells growth and metastasis: implication of Wnt/catenin beta and MEK/ERK signaling pathways" was retracted in 2024. Reasons: duplicated images; unreliable results or conclusions; concerns about the data.

Non coding RNAs, including long non coding RNAs and short non coding RNAs, are proved to involve in many biology of normal and cancer cells [32, 33]. Short non coding RNAs contain microRNAs (miRNAs), small interference RNAs (siRNAs) and PIWI protein binding RNAs (piRNAs) [34]. MiRNAs could play crucial roles as oncogene or antioncogene in human cancers. MiRNAs regulated cancer related growth, metabolism, genomic stability, apoptosis, epithelial to mesenchymal transition (EMT), tumor cell microenvironment and angiogenesis have been well demonstrated [35, 36]. Recently, decreased levels of miR-338-3p were observed in breast cancer, gastric cancer and esophageal squamous cell carcinoma compared to normal tissues, positively related with overall survival, and could serve as a poor prognostic marker, which indicated miR-338-3p might play as tumor suppressor in those malignant tumors [37–39]. Our previous report indicated miR-338-3p was downregulated in epithelial ovarian cancer tissues and was negatively correlated with MACC1 expression [14], but those results were observed from small enrolled patient numbers and single center cohort study. Thence, expression profile of miR-338-3p in ovarian cancer tissues still needs to be confirmed by other independent researches with large enrolled patient numbers. In present study, biomedical databases containing different independent cohorts with large enrolled patient numbers were queried to confirm the expression profile of miR-338-3p in ovarian cancer tissues. In the other hand, we also detected lower levels of miR-338-3p in ovarian cancer cells than normal ovary cells, which also were confirmed by other two independent studies [12, 13]. Therefore, the expression profiles of miR-338-3p in ovarian cancer tissues and cancer cells were all downregulated, which indicated miR-338-3p might play an antitumor role in ovarian cancer.

Commonly, miRNAs were considered to bind to downstream target genes and inhibit gene transcription or induce gene degradation [40]. Multiply biomedical databases query and previous reports showed miR-338-3p could directly bind to MACC1 and inhibit MACC1 in different human cancer cells, which also was confirmed in present study by dual-luciferase reporter assay and western blot assay in ovarian cancer cells. Those results indicated that miR-338-3p could bind to and regulate MACC1 gene in ovarian cancer cells.

The article "MicroRNA-338-3p suppresses ovarian cancer cells growth and metastasis: implication of Wnt/catenin beta and MEK/ERK signaling pathways" was retracted in 2024. Reasons: duplicated images; unreliable results or conclusions; concerns about the data.

To examine the effects of miR-338-3p on the growth and metastasis of ovarian cancer cells, we overexpressed miR-338-3p in ovarian cancer OVCAR3 and OVCAR8 cells. Inhibition of proliferation, migration and invasion were observed following miR-338-3p restoration in vitro, which indicated miR-338-3p could suppress the growth and metastasis of ovarian cancer cells in vitro.

To explore the possible mechanism underlying miR-338-3p regulated growth and metastasis of ovarian cancer cells, we focused on MACC1, Met and its downstream signaling pathway. MACC1 were closely related to the invasion and metastasis, could be used as a prognostic marker for advanced colon cancer, gastric cancer, lung cancer and hepatocellular carcinoma, which also was proved in our previous reports in ovarian cancer [41–45]. MACC1 can regulate the expression of Met by binding to the sp1 site, which is about 60 bp upstream of the MET gene promoter [46, 47]. Met is the key factor of HGF/Met signaling, which is the most important regulator of EMT [48]. HGF/Met signaling can induce stromal cells to disrupt cell-cell junctions, expose extracellular matrix, and promote growth, adhesion, migration, invasion and vascular endothelial cell growth of various malignant tumor cells, including ovarian cancer [49]. We found that MACC1 and Met was downregulated after miR-338-3p restoration, and miR-338-3p could attenuate the proliferation, migration and invasion induced by MACC1 or Met overexpression in present study, which might due to the inhibition of MACC1 by miR-338-3p and direct regulation of Met by miR-338-3p.

EMT can reduce the adhesion between cells and increase cells motility and invasiveness, and EMT also is demonstrated to paly crucial roles in the invasion and metastasis of ovarian cancer and many other human cancers [50]. Human cancer related EMT is characterized with upregulation of the enzymes that decompose the extracellular matrix (such as MMPs) and mesenchymal markers (including Vimentin, Catenin beta and N-cadherin), and downregulation of epithelial markers (including E-cadherin and Cytokeratin7) [51]. PCNA usually serves as a canonical proliferation marker. Furthermore, downregulation of E-cadherin is considered as a hallmark of EMT [52]. Following restoration of miR-338-3p, PCNA, MMP2, MMP9, N-cadherin, Catenin beta and Vimentin were decreased, while E-cadherin and Cytokeratin7 were increased shown in our present data. MACC1 and Met overexpression induced upregulation of PCNA, MMP2, MMP9, N-cadherin, Catenin beta and Vimentin and downregulation of E-cadherin and Cytokeratin7 could be reversed by miR-338-3p, at least in partially. These data indicated that overexpression of miR-338-3p could suppress the proliferation and EMT induced by MACC1 and Met overexpression in ovarian cancer cells.

The article "MicroRNA-338-3p suppresses ovarian cancer cells growth and metastasis: implication of Wnt/catenin beta and MEK/ERK signaling pathways" was retracted in 2024. Reasons: duplicated images; unreliable results or conclusions; concerns about the data.

Malignant growth and metastasis involve in many intricate and detailed signaling transductions in cancer cells. Once Met is activated, it can transmit extracellular signals to activate many intracellular pathways, including MAPK, EGFR, VEGF and PI3K signaling pathways, and participate in many physiological and pathological processes such as cell proliferation, apoptosis, migration and invasion [53]. We previously reported MACC1 might regulate MEK/ERK pathway to involve in the invasion and metastasis of ovarian cancer cells [41]. Aberrant activation of canonical Wnt/Catenin beta pathway was also closely related with the proliferation, differentiation, motility, invasion and metastasis of normal and malignant tumor cells [54]. Wnt3a as a Wnt ligand is a main member of Wnt family, and p-LRP6 function as co-receptors for Wnt family and are required for the activation of canonical Wnt/Catenin beta signaling pathway [55]. Besides the KEGG pathway analysis results, our western blot data also showed expressions of Catenin beta and activities of Wnt/Catenin beta and MEK/ERK pathways in ovarian cancer cells, as well as MACC1 or Met upregulation induced expressions of Catenin beta and activities of Wnt/Catenin beta and MEK/ERK pathways in ovarian cancer cells, could be suppressed by miR-338-3p upregulation, which indicated that miR-338-3p could attenuate MACC1 or Met induced Wnt/Catenin beta and MEK/ERK signaling activities in ovarian cancer cells.

We also using xenograft mouse model to confirm the data explored in vitro. Upregulation of miR-338-3p could inhibit the xenograft tumor growth and metastasis in vivo. Decreased PCNA, MMP2, MMP9, Vimentin, Catenin beta and N-cadherin, increased E-cadherin and Cytokeratin7, and decreased activities of Wnt/Catenin beta and MEK/ERK pathways could be detected in miR-338-3p overexpression lentivectors transfected xenograft tumor tissues. These data indicated miR-338-3p could suppress the growth and metastasis of ovarian cancer cells via MACC1 and Met regulated Wnt/Catenin beta and MEK/ERK pathways in vivo.

## Conclusions

Taken together, using database query and in vivo and in vitro assay, our study showed restoration of miR-338-3p could suppress the growth and metastasis of ovarian cancer cells in vitro and in vivo, which was implicated in MACC1 and Met regulated Wnt/Catenin beta and MEK/ERK pathways. and oOur data might be helpful to elaborate the complicate molecular mechanisms and explore new therapy strategies for the ovarian cancer. However, the present study only investigated few parts of the regulation mechanisms of ovarian cancer malignant behaviors, further studies about the relations between miRNAs and malignant growth and metastasis of ovarian cancer still need to be performed.

The article "MicroRNA-338-3p suppresses ovarian cancer cells growth and metastasis: implication of Wnt/catenin beta and MEK/ERK signaling pathways" was retracted in 2024. Reasons: duplicated images; unreliable results or conclusions; concerns about the data.

## Supplementary information

**Additional file 1.** KEGG Pathways Enrichment Analysis results.

**Additional file 2.** Target genes of miR-338-3p predicted by biomedical database.

## Data Availability

The databases queried and/or analyzed in the present study are available in dbDEMC (www.picb.ac.cn/dbDEMC/index.html), cBioPortal (https://www.cbioportal.org/), OncomiR (http://www.oncomir.org/), TargetScan Human (http://www.targetscan.org/vert_72/), miRpathDB (https://mpd.bioinf.uni-sb.de/), microT-CDS (http://diana.imis.athena-innovation.gr/DianaTools/index.php?r=microT_CDS/index), miRTarBase (http://mirtarbase.mbc.nctu.edu.tw/php/index.php), miRTargetLink (https://ccb-web.cs.uni-saarland.de/mirtargetlink/) and ENCORI (http://starbase.sysu.edu.cn/) online websites.

## Abbreviations

ATCC: American Type Culture Collection
CCTCC: China Center for Type Culture Collection
EMT: Epithelial to mesenchymal transition
FBS: Fetal bovine serum
GAPDH: Glyceraldehyde 3-phosphate dehydrogenase
KEGG: Kyoto Encyclopedia of Genes and Genomes
MACC1: MET transcriptional regulator MACC1
miR-338-3p: MicroRNA-338-3p
PCNA: Proliferating cell nuclear antigen
UTRs: Untranslated regions

## References

[1] Hanahan D, Weinberg RA (2011). Hallmarks of cancer: the next generation. Cell.

[2] Konecny GE, Winterhoff B, Kolarova T, Qi J, Manivong K, Dering J (2011). Expression of p16 and retinoblastoma determines response to CDK4/6 inhibition in ovarian cancer. Clin Cancer Res.

[3] Hamanishi J, Mandai M, Ikeda T, Minami M, Kawaguchi A, Murayama T (2015). Safety and antitumor activity of anti-PD-1 antibody, Nivolumab, in patients with platinum-resistant ovarian Cancer. J Clin Oncol.

[4] Dizon DS (2017). PARP inhibitors for targeted treatment in ovarian cancer. Lancet.

[5] Siegel RL, Miller KD, Jemal A (2019). Cancer statistics, 2019. CA Cancer J Clin.

[6] Mendell JT (2005). MicroRNAs: critical regulators of development, cellular physiology and malignancy. Cell Cycle.

[7] Gaedcke J, Grade M, Camps J, Sokilde R, Kaczkowski B, Schetter AJ (2012). The rectal Cancer microRNAome - microRNA expression in rectal Cancer and matched Normal mucosa. Clin Cancer Res.

The article "MicroRNA-338-3p suppresses ovarian cancer cells growth and metastasis: implication of Wnt/catenin beta and MEK/ERK signaling pathways" was retracted in 2024. Reasons: duplicated images; unreliable results or conclusions; concerns about the data.

[8] Guo B, Liu LY, Yao JY, Ma RL, Chang DM, Li ZF (2014). miR-338-3p suppresses gastric Cancer progression through a PTEN-AKT Axis by targeting P-REX2a. Mol Cancer Res.

[9] Liu J, Cao LG, Zhao N, Feng Y, Yu Z, Li YH (2019). miR-338-3p inhibits A549 lung cancer cell proliferation and invasion by targeting AKT and beta-catenin signaling pathways. Mol Med Rep.

[10] Chen X, Pan M, Han LL, Lu HT, Hao XW, Dong Q (2013). miR-338-3p suppresses neuroblastoma proliferation, invasion and migration through targeting PREX2a. FEBS Lett.

[11] Zhang T, Liu W, Zeng XC, Jiang N, Fu BS, Guo Y (2016). Down-regulation of microRNA-338-3p promoted angiogenesis in hepatocellular carcinoma. Biomed Pharmacother.

[12] Zhang Y, Shi B, Chen J, Hu L, Zhao C (2016). MiR-338-3p targets pyruvate kinase M2 and affects cell proliferation and metabolism of ovarian cancer. Am J Transl Res.

[13] Wen C, Liu X, Ma H, Zhang W, Li H (2015). MiR3383p suppresses tumor growth of ovarian epithelial carcinoma by targeting Runx2. Int J Oncol.

[14] Zhang R, Shi H, Ren F, Liu Z, Ji P, Zhang W (2019). Down-regulation of miR-338-3p and up-regulation of MACC1 indicated poor prognosis of epithelial ovarian Cancer patients. J Cancer.

[15] Yang Z, Wu L, Wang A, Tang W, Zhao Y, Zhao H (2017). dbDEMC 2.0: updated database of differentially expressed miRNAs in human cancers. Nucleic Acids Res.

[16] Gao J., Aksoy B. A., Dogrusoz U., Dresdner G., Gross B., Sumer S. O., Sun Y., Jacobsen A., Sinha R., Larsson E., Cerami E., Sander C., Schultz N. (2013). Integrative Analysis of Complex Cancer Genomics and Clinical Profiles Using the cBioPortal. Science Signaling.

[17] Wong NW, Chen YH, Chen S, Wang XW (2018). OncomiR: an online resource for exploring pan-cancer microRNA dysregulation. Bioinform.

[18] Hamberg Maarten, Backes Christina, Fehlmann Tobias, Hart Martin, Meder Benjamin, Meese Eckart, Keller Andreas (2016). miRTargetLink—miRNAs, Genes and Interaction Networks. International Journal of Molecular Sciences.

[19] Lewis BP, Burge CB, Bartel DP (2005). Conserved seed pairing, often flanked by adenosines, indicates that thousands of human genes are microRNA targets. Cell.

[20] Paraskevopoulou MD, Georgakilas G, Kostoulas N, Vlachos IS, Vergoulis T, Reczko M (2013). DIANA-microT web server v5.0: service integration into miRNA functional analysis workflows. Nucleic Acids Res.

[21] Backes C, Kehl T, Stockel D, Fehlmann T, Schneider L, Meese E (2017). miRPathDB: a new dictionary on microRNAs and target pathways. Nucleic Acids Res.

[22] Chou CH, Shrestha S, Yang CD, Chang NW, Lin YL, Liao KW (2018). miRTarBase update 2018: a resource for experimentally validated microRNA-target interactions. Nucleic Acids Res.

The article "MicroRNA-338-3p suppresses ovarian cancer cells growth and metastasis: implication of Wnt/catenin beta and MEK/ERK signaling pathways" was retracted in 2024. Reasons: duplicated images; unreliable results or conclusions; concerns about the data.

[23] Zhang RT, Shi HR, Ren F, Liu HN, Zhang MH, Deng YX (2015). Misregulation of polo-like protein kinase 1, P53 and P21(WAF1) in epithelial ovarian cancer suggests poor prognosis. Oncol Rep.

[24] Huang Na, Wu Zhenzhen, Zhou Minyu, Wang Lin, Ma Huanrong, Shi Min, Zuo Qiang, Zheng Dayong, Liao Wangjun (2014). Effect of MiR-338-3p on epithelial-mesenchymal transition in gastric cancer cells by targeting ZEB2 and MACC1 and regulation of MACC1/c-Met signaling. Journal of Clinical Oncology.

[25] Shang C, Hong Y, Guo Y, Xue YX. Mir-338-3p inhibits malignant biological behaviors of Glioma cells by targeting MACC1 gene. Med Sci Monitor. 2016;22:710–6.10.12659/MSM.897055PMC478027026936749

[26] Zou T, Duan J, Liang JT, Shi HJ, Zhen TT, Li H (2018). miR-338-3p suppresses colorectal cancer proliferation and progression by inhibiting MACC1. Int J Clin Exp Patho.

[27] Lu ML, Huang H, Yang JH, Li J, Zhao GF, Li WH (2019). miR-338-3p regulates the proliferation, apoptosis and migration of SW480 cells by targeting MACC1. Exp Ther Med.

[28] Zhang CH, Li H, Wang JL, Zhang JB, Hou XQ (2019). MicroRNA-338-3p suppresses cell proliferation, migration and invasion in human malignant melanoma by targeting MACC1. Exp Ther Med.

[29] Hua FF, Liu SS, Zhu LH, Wang YH, Liang X, Ma N (2017). MiRNA-338-3p regulates cervical cancer cells proliferation by targeting MACC1 through MAPK signaling pathway. Eur Rev Med Pharmaco.

[30] Jessmon P, Boulanger T, Zhou W, Patwardhan P (2017). Epidemiology and treatment patterns of epithelial ovarian cancer. Expert Rev Anticanc.

[31] Eisenhauer EA (2017). Real-world evidence in the treatment of ovarian cancer. Ann Oncol.

[32] Adelman K, Egan E (2017). NON-CODING RNA more uses for genomic junk. Nat.

[33] Anastasiadou E, Jacob LS, Slack FJ (2018). Non-coding RNA networks in cancer. Nat Rev Cancer.

[34] Ghildiyal M, Zamore PD (2009). Small silencing RNAs: an expanding universe. Nat Rev Genet.

[35] Iorio MV, Croce CM (2012). microRNA involvement in human cancer. Carcinog.

[36] Slaby O, Laga R, Sedlacek O (2017). Therapeutic targeting of non-coding RNAs in cancer. Biochem J.

[37] Vivacqua Adele, Sebastiani Anna, Miglietta Anna, Rigiracciolo Damiano, Cirillo Francesca, Galli Giulia, Talia Marianna, Santolla Maria, Lappano Rosamaria, Giordano Francesca, Panno Maria, Maggiolini Marcello (2018). miR-338-3p Is Regulated by Estrogens through GPER in Breast Cancer Cells and Cancer-Associated Fibroblasts (CAFs). Cells.

[38] Liu S, Suo J, Wang C, Sun X, Wang D, He L (2017). Downregulation of tissue miR-338-3p predicts unfavorable prognosis of gastric cancer. Cancer Biomark.

The article "MicroRNA-338-3p suppresses ovarian cancer cells growth and metastasis: implication of Wnt/catenin beta and MEK/ERK signaling pathways" was retracted in 2024. Reasons: duplicated images; unreliable results or conclusions; concerns about the data.

[39] Li X, Li Z, Yang G, Pan Z (2015). MicroRNA-338-3p suppresses tumor growth of esophageal squamous cell carcinoma in vitro and in vivo. Mol Med Rep.

[40] Zamore PD, Haley B (2005). Ribo-gnome: the big world of small RNAs. Sci.

[41] Zhang Ruitao, Shi Huirong, Chen Zhimin, Wu Qinghua, Ren Fang, Huang Haoliang (2011). Effects of metastasis-associated in colon cancer 1 inhibition by small hairpin RNA on ovarian carcinoma OVCAR-3 cells. Journal of Experimental & Clinical Cancer Research.

[42] Shirahata A, Shinmura K, Kitamura Y, Sakuraba K, Yokomizo K, Goto T (2010). MACC1 as a marker for advanced colorectal carcinoma. Anticancer Res.

[43] Shirahata A, Sakata M, Kitamura Y, Sakuraba K, Yokomizo K, Goto T (2010). MACC 1 as a marker for peritoneal-disseminated gastric carcinoma. Anticancer Res.

[44] Shirahata A, Fan W, Sakuraba K, Yokomizo K, Goto T, Mizukami H (2011). MACC 1 as a marker for vascular invasive hepatocellular carcinoma. Anticancer Res.

[45] Shimokawa H, Uramoto H, Onitsuka T, Gu CD, Hanagiri T, Oyama T (2011). Overexpression of MACC1 mRNA in lung adenocarcinoma is associated with postoperative recurrence. J Thorac Cardiov Sur.

[46] Stein U, Smith J, Walther W, Arlt F (2009). MACC1 controls met what a difference an Sp1 site makes. Cell Cycle.

[47] Kokoszynska K, Krynski J, Rychlewski L, Wyrwicz LAS (2009). Unexpected domain composition of MACC1 links MET signaling and apoptosis. Acta Biochim Pol.

[48] Tsarfaty I, Rong S, Resau JH, Rulong S, da Silva PP, Vande Woude GF (1994). The met proto-oncogene mesenchymal to epithelial cell conversion. Science..

[49] Zhou HY, Pon YL, Wong AS (2008). HGF/MET signaling in ovarian cancer. Curr Mol Med.

[50] Huang RY, Chung VY, Thiery JP (2012). Targeting pathways contributing to epithelial-mesenchymal transition (EMT) in epithelial ovarian cancer. Curr Drug Targets.

[51] Thiery JP (2003). Epithelial-mesenchymal transitions in development and pathologies. Curr Opin Cell Biol.

[52] Gotzmann J, Mikula M, Eger A, Schulte-Hermann R, Foisner R, Beug H (2004). Molecular aspects of epithelial cell plasticity: implications for local tumor invasion and metastasis. Mutat Res.

[53] Potempa S, Ridley AJ (1998). Activation of both MAP kinase and phosphatidylinositide 3-kinase by Ras is required for hepatocyte growth factor scatter factor-induced adherens junction disassembly. Mol Biol Cell.

[54] Logan CY, Nusse R (2004). The Wnt signaling pathway in development and disease. Annu Rev Cell Dev Biol.

[55] Tamai K, Semenov M, Kato Y, Spokony R, Liu C, Katsuyama Y (2000). LDL-receptor-related proteins in Wnt signal transduction. Nat.

